# An Occult Hepatitis B-Derived Hepatoma Cell Line Carrying Persistent Nuclear Viral DNA and Permissive for Exogenous Hepatitis B Virus Infection

This article has been retracted.

**DOI:** 10.1371/journal.pone.0065456

**Published:** 2013-05-29

**Authors:** Chih-Lang Lin, Rong-Nan Chien, Shi-Ming Lin, Po-Yuan Ke, Chen-Chun Lin, Chau-Ting Yeh

**Affiliations:** 1 Liver Research Unit, Chang Gung Memorial Hospital and Chang Gung University College of Medicine, Keelung, Taiwan; 2 Graduate Institute of Clinical Medical Sciences, College of Medicine, Chang Gung University, Taoyuan, Taiwan; 3 Liver Research Center, Chang Gung Memorial Hospital, Taipei, Taiwan; 4 Department of Biochemistry and Molecular Biology, Chang Gung University, Taoyuan, Taiwan; The University of Hong Kong, Hong Kong

## Abstract

Occult hepatitis B virus (HBV) infection is defined as persistence of HBV DNA in liver tissues, with or without detectability of HBV DNA in the serum, in individuals with negative serum HBV surface antigen (HBsAg). Despite accumulating evidence suggesting its important clinical roles, the molecular and virological basis of occult hepatitis B remains unclear. In an attempt to establish new hepatoma cell lines, we achieved a new cell line derived from a hepatoma patient with chronic hepatitis C virus (HCV) and occult HBV infection. Characterization of this cell line revealed previously unrecognized properties. Two novel human hepatoma cell lines were established. Hep-Y1 was derived from a male hepatoma patient negative for HCV and HBV infection. Hep-Y2 was derived from a female hepatoma patient suffering from chronic HCV and occult HBV infection. Morphological, cytogenetic and functional studies were performed. Permissiveness to HBV infection was assessed. Both cell lines showed typical hepatocyte-like morphology under phase-contrast and electron microscopy and expressed alpha-fetoprotein, albumin, transferrin, and aldolase B. Cytogenetic analysis revealed extensive chromosomal anomalies. An extrachromosomal form of HBV DNA persisted in the nuclear fraction of Hep-Y2 cells, while no HBsAg was detected in the medium. After treated with 2% dimethyl sulfoxide, both cell lines were permissive for exogenous HBV infection with transient elevation of the replication intermediates in the cytosol with detectable viral antigens by immunoflurescence analysis. In conclusions, we established two new hepatoma cell lines including one from occult HBV infection (Hep-Y2). Both cell lines were permissive for HBV infection. Additionally, Hep-Y2 cells carried persistent extrachromosomal HBV DNA in the nuclei. This cell line could serve as a useful tool to establish the molecular and virological basis of occult HBV infection.

## Introduction

Chronic hepatitis B virus (HBV) infection is one of the major infectious diseases worldwide and may lead to severe liver diseases, including liver cirrhosis and hepatocellular carcinoma (HCC) [1], [2]. HBV is a small, enveloped partially double-stranded DNA virus of the family *Hepadnaviridae*, which replicates via reverse transcription. The 3.2-kb relaxed circular DNA (RC-DNA) genome encapsidated by the viral particles is transported into the host cell nuclei, where it is repaired to become covalently closed circular DNA (cccDNA)—the template for transcription of several subgenomic and genomic RNAs [3]. Much has been learned about HBV host–pathogen interactions since its discovery, but many unsolved issues remain, such as the mechanism of viral entry, the exact role of some viral components, the kinetics of HBV cccDNA production, and the precise mechanism that leads to the development of HCC [4].

A prime characteristic of HBV is that it exhibits a very narrow host range and a strong tropism for liver parenchymal cells [5], [6]. To investigate the complete life cycle of HBV infection—despite the usefulness of available human liver cell lines—there is clearly a strong need for appropriate in vitro infection systems, allowing for exogenous HBV infection [7]. HBV replication can be initiated by genomic DNA transfection into HepG2, Huh7, HepAD38, or primary hepatocytes [8]. However, until recent years, exogenous HBV infection has only been successfully achieved using primary human hepatocytes [9], [10]. However, the system is limited by a low susceptibility to infection and the cultured hepatocytes become non-permissive for HBV soon after plating. Until now, highly efficient HBV infection is accomplished in only one well differentiated hepatoma cell line (Hepa RG) established from a female patient suffering from HCC and hepatitis C virus (HCV) infection [5]. As such, establishment of new HBV permissive human hepatoma cell lines for the study of HBV biology and the development of new anti-HBV strategy is needed.

The persistence of HBV genomes in the blood or liver of individuals negative for HBV surface antigen (HBsAg) is termed occult HBV infection [11]. It is not known why occult HBV carriers are HBsAg-negative. Some of these individuals are infected by viral variants that either produce an antigenically modified HBV surface protein—undetectable by even the most sensitive available HBsAg assays—or carry mutations capable of inhibiting surface protein gene expression and/or viral replication [12]. However, such mutations cannot be detected in a large proportion of occult hepatitis B patients. Several other hypotheses have been raised for the molecular mechanisms of occult hepatitis B infection, including HBV infection in host mononuclear cells and formation of immune complex interfering HBsAg detection. Experimental evidences are still in need to determine whether one or some of them stands.

Substantial clues indicate that occult HBV infection is associated with the progression of liver fibrosis and cirrhosis development [11], [13], [14], and that it is a risk factor for HCC development [15], [16] in patients with cryptogenic liver disease. Several reports performed in the 1990s suggested that occult HBV may negatively influence chronic HCV infection by reducing the response to IFN therapy [17], [18], [19]. Thus, there is a strong need to establish appropriate cell-based systems to study the molecular mechanism of occult HBV infection. To our knowledge, cell culture systems derived from patients with occult HBV infection, capable of maintaining sustained HBV replication, have not yet been generated.

In this study, we established 2 hepatoma cell lines which expressed a representative panel of liver-specific proteins and were susceptible to exogenous HBV infection. Notably, we produced the first stable hepatoma cell line derived from occult hepatitis B patient, wherein a nuclear form of HBV DNA persisted during multiple cell line passages without secretion of HBsAg. This cell line provides a novel tool suitable for studying several important aspects of occult HBV infection.

## Materials and Methods

### Cell line establishment and culture conditions

This study was approved by the Institutional Review Board of Chang Gung Medical Center. Hep-Y1 cells were grown from the fine-needle-aspirated hepatoma cells of a male patient suffering from HCC without HBV and HCV infection. Hep-Y2 cells were isolated from the fine-needle-aspirated hepatoma cells of a female patient suffering from HCC with occult HBV and chronic HCV infection. Occult HBV infection is defined as persistence of viral genomes in the blood or liver of individuals negative for HBsAg. Chronic HCV infection is defined as seropositive for anti-HCV antibodies and HCV RNA for more than 6 months.

HCC cells were aspirated under echo-guided procedure using a fine needle at the same time when aspiration cytology was needed for diagnosis. Human methothelial cells were isolated from ascites of cirrhotic patients and plated as a confluent monolayer in culture dishes. HCC cells were seeded on to the methothelial cells and incubated at 37°C in a humidified atmosphere containing 5% CO_2_ and 95% air. The cells were grown in a 1∶1 mixture of RPMI-1640 medium (Gibco, Invitrogen Corporation, Carlsbad, CA) and PromoCell Hepatocyte Medium (PromoCell GmbH, Heidelberg, Germany) supplemented with 2 mM l-glutamine, 10 mM HEPES buffer, 10% heat-inactivated fetal bovine serum (FBS), 100 U/mL penicillin, 100 µg/mL streptomycin, and 0.25 µg/mL amphotericin B. The cells were trypsinized and re-plated every 7 days, allowing for senescence and death of methothelial cells. After 5 passages, the cells were grown in only RPMI-1640 medium with supplements. After >20 passages, the cultured cells, if still growing, were collected and stored in liquid nitrogen [20].

### Serological assays, HBV DNA assay, and HCV RNA assay

HBsAg was measured by an enzyme immunoassay (Enzygnost HBsAg 5.0; Dade Behring Marburg GmbH, Marburg, Germany) and a radioimmunoassay (Ausria-II; Abbott, Abbott Park, IL). Serum antibody to HCV was assayed using commercially available second- or third-generation enzyme immunoassay kits (HCV EIA II or III; Abbott Laboratories). Serum HBV DNA levels were quantified using a COBAS TaqMan HBV test (Roche Molecular Systems, Inc., Pleasanton, CA) with a detection limit of 68 copies/mL. In this test, 5.82 copies/mL was equivalent to 1 IU/mL. HCV RNA in the serum sample and in the culture medium was assessed by use of a COBAS TaqMan HCV test (Roche Molecular Systems, Inc., Pleasanton, CA). Quantification of HBsAg was performed using Elecsys HBsAg II assay (Roche Diagnostic).

Two HCC cell lines were described in this report. Hep-Y1 cells were derived from a HCC patient with negative anti-HCV antibody and negative HBsAg. HCV RNA was negative in both the serum sample of this patient and the culture medium of Hep-Y1 cells. Hep-Y2 was derived from a HCC patient with positive anti-HCV antibody. In this patient, the serum HCV RNA level was 12444 IU/mL. However, in the culture medium of Hep-Y2 cells, HCV RNA was negative. In the Hep-Y2-derived patient, the serum HBV DNA level was negative immediately and 6 months after the fine needle aspiration procedure. However, HBV DNA was positive in the liver tissue by PCR assay, which is in concordance with the definition of occult HBV infection [12].

### HBV infection in cell lines

Hep-Y1cells and Hep-Y2 cells were grown on coverslips with RPMI-1640 medium at 37°C in 5% CO2 air. At 24 h after plating, Hep-Y1cells and Hep-Y2 cells were inoculated with 500 µL of HBV-positive serum (4.2×10 ^9^ copies/mL and 3.2 × 10 ^9^ copies/mL, respectively). In control group, HBV-negative serum was used. During the inoculation, cells were maintained in the presence of 2% dimethyl sulfonxide (DMSO) and harvested at the indicated time-points.

### Extraction of HBV DNA and polymerase chain reaction (PCR)

To isolate HBV DNA, viral replicative DNA intermediates were isolated from whole cell lysates. Cells were trypsinized and separated into nuclear and cytoplasmic fractions using cell lysis buffer (100 mM Tris-HCl [pH 7.4], 0.5% NP40, and 150 mM NaCl). DNA in the nucleus was further partitioned by the Hirt (1% SDS, 10 mM EDTA, 5 mM EGTA [pH 7.5], and 1 M NaCl) procedure into supernatant (extrachromosome) and pellet (chromosome) fractions. Cytoplasmic and nuclear extrachromosomal fractions were mixed with TEN buffer (1 M Tris-HCl [pH 7.5], 0.5 M EDTA [pH 8.0], 5 M NaCl, and 10% SDS) supplemented with proteinase K (1 mg/ml) and incubated at 55°C for 3 hr. For HBV DNA extraction from the serum and culture medium, 100 µL sample was mixed with 300 µL of buffer (13.3 mM Tris-HCl, pH 8.0, 6.7 mM EDTA, 0.67% SDS and 133 mg/mL proteinase K) and incubated at 55°C for 4 h. Two phenol/chloroform extractions were followed by one chloroform extraction, and DNA was precipitated with cold ethanol. The precipitate was dissolved in TE buffer (10 mM Tis-HCl [pH 8.0] and 1 mM EDTA). PCR was performed with 10 µL of DNA, 2 units of Super Tag (HT Biotechnology, Cambridge, UK), 200 µmol/L deoxynucleotide triphosphate, 100 pmol of each primer, and the reaction buffer that was provided with the enzyme. The PCR primers used were as follows: 5′-CTTATTGGTTCTTCTGGATTATC-3′ (P1, nt. 433–455, sense) and 5′-GTTTAAATGTATACCCAGAGAC-3′ (P2, nt. 837–816, antisense) [21]. The program cycle consisted of 94°C for 1 min, 55°C for 1 min, and 72°C for 1 min. Amplification proceeded for 30 cycles in a thermal cycler (Perkin-Elmer Cetus, Norwalk, CT). A serum sample from a normal subject and an aliquot of water were included as negative controls. Nucleic acids were analyzed on a 2% agarose gel. The sensitivity and specificity of the aforementioned assays were previously tested according to the methods of Liaw et al [2].

### Southern and western blot analyses

The sequence flanked by primers P1 and P2 was amplified, labeled, and used as the probe for Southern blot analysis. The detailed methods for probe labeling and Southern blotting have previously been described [22]. The medium (100 µL) from the cell culture plates was loaded directly onto the nitrocellulose membrane. The following antibodies (1∶1000 dilution) were tested: albumin polyclonal antibody (lot A80–129A; Bethyl Laboratories, Montgomery, TX), aldolase B monoclonal antibody (lot GTX62246; GeneTex, Irvine, CA), and transferrin polyclonal antibody (lot GTX112729; GeneTex). To perform sodium dodecyl sulfate–polyacrylamide gel electrophoresis, cells were lysed in Tris-buffered saline (TBS) (10 mmol/L Tris-HCl [pH 7.2], 150 mmol/L NaCl) containing 0.5% Nonidet P-40 (Sigma Chemical Co., St. Louis, MO) and were centrifuged at 1500 *g*. Both the soluble (cytoplasmic) fraction and the culture medium were subjected to SDS–PAGE, followed by western blot analysis. As a control, GAPDH was detected by the use of anti-GAPDH antibody (6C5; Novus Biologicals, Littleton, CO).

### Immunofluorescence analysis

Hep-Y1cells and Hep-Y2 cells were grown on coverslips and infected using 500 ul of HBV-positive serum (4.2 × 10 ^9^ copies/mL and 3.2 × 10 ^9^ copies/mL). Forty-eight hours post-transfection, the cells were fixed in acetone at −20°C for 2 min. Rabbit polyclonal anti-HBs and anti-HBc antibody (ViroStat; 1∶100 dilution) and fluorescein isothiocyanate-conjugated goat anti-rabbit antibody (Leinco Technologies, Inc., St. Louis, MO; 1∶150 dilution) were used as the primary and secondary antibodies, respectively. To visualize the nuclei, cells were stained with 4′,6-diamidino-2-phenylindole (DAPI; 200 ng/mL).

### Chromosome preparation and cytogenetic analysis

Standard Giemsa-banded karyotype analysis was performed according to the manufacturer's instructions, with modifications as previously described [20]. Briefly, after standard culturing of cell lines, chromosome spreads were prepared for performing karyotype analysis. The cells were then treated with hypotonic solution (0.1 M MgCl_2_), fixed with Carnoy's acetic solution, and stained with 0.8% Giemsa solution. The clonality criteria and the karyotype description followed the recommendations of the International System for Human Cytogenetic Nomenclature (ISCN) [23].

## Results

### Morphology of the cell lines

Morphological assessment of both Hep-Y1 and Hep-Y2 (Figure 1A) cells by phase-contrast microscopy revealed a typical monolayer of bright and spherically shaped cells with characteristic well-contrasted borders. The majority of cells adhered to each other, presenting with a fascicular pattern of growth and granular hepatocyte-like appearance. Binuclei were observed in the majority of cells, the hepatic plate-like structures were noted, and the boundaries between hepatocytes were perfectly clear and bright. The presumably bile canaliculi and sinusoidal complexes were vague, and short microvilli were scattered over the plasma membrane surface.

**Figure 1:** Phase-contrast and transmission electron micrographs under proliferating conditions. (A) Morphology of Hep-Y1 and Hep-Y2 cells in monolayer culture by phase-contrast microscopy. Cells were maintained in RPMI-1640 medium. Arrows indicated granular hepatocyte-like appearance. Arrowheads indicated hepatic plate-like structure. (B) Low- magnification views of a single Hep-Y2 cell by transmission electron microscopy. Arrows indicated prominent nucleoli. Arrowheads indicated mitochondria. (C) High-magnification views of a single Hep-Y2 cell by transmission electron microscopy. Arrowheads indicated mitochondria. (D) Low- magnification views of a single Hep-Y1 cell by transmission electron microscopy. Arrows indicated prominent nucleoli. Arrowheads indicated mitochondria. (E) High-magnification views of a single Hep-Y1 cell by transmission electron microscopy. Arrowheads indicated mitochondria.

Transmission electron microscopy of Hep-Y2 cells (Figure 1A, B, and C) and Hep-Y1 cells (Figure 1A, D and E) demonstrated normal hepatocyte subcellular architecture with plentiful mitochondria. In addition, endoplasmic reticulum and Golgi; nuclei with prominent nucleoli; and well-defined nuclear pores, lipid vacuoles, and pools of glycogen were observed. Structures identical to bile canaliculi were also delineated by typical junctional complexes and presented with microvilli (Figure 1C and 1E).

### Cytogenetic studies

Cytogenetic studies by standard Giemsa-banded karyotype analysis showed both structural and chromosomal abnormalities (Figure 2). Consistent with the findings of DNA content, the karyotype results of Hep-Y1 and Hep-Y2 cells revealed aneuploidy, presenting with 75, XX <3N> and 57, X <2N>, respectively. Complicated genetic abnormalities of chromosomal structure in Hep-Y1 cells, including +del(1)(p13), +der(1)t(1;?)(q10;?), add(2)(p23), +i(8)(q10), add(9)(p24), der(15;17)(q10;q10), +del(16)(q22), and +add(17)(p11.2) were observed. Among analyzed cells, chromosome gains, involving chromosomes 3, 7, 20, and 22, and chromosome losses, involving chromosomes 4, 5, 6, 9, 15, 18, and 21, and additional 5 marker chromosomes were noted in Hep-Y1 cells. The genetic abnormalities seen in Hep-Y2 cells were del(1)(q10), der(2)t(2;?)(p23;?), der(3)t(3;?)(p11;?), +i(7)(q10), +der(7)t(7;?)(q11.2;?), der(11)t(1;11)(q23;q23), and +ass(19)(q13.4). Among analyzed cells, chromosome number alterations of chromosomes in Hep-Y2 cells comprised gains in chromosomes 6, 14, 15, and 20, and losses on chromosome 17, and 5 marker chromosomes.

**Figure 2:** Standard Giemsa-banded karyotype analysis. Representative chromosomal structures of Hep-Y1 cell (A) and Hep-Y2 cell (B) displayed aneuploidy and complicated genetic abnormalities. Arrows indicated chromosome gains. Arrowheads indicated marker chromosomes.

### Expression of liver-specific functions

To further determine the liver-specific functional competencies of Hep-Y1 and Hep-Y2 cells, we subsequently tested for the secretion of alpha-fetoprotein (AFP) and cellular expression of albumin, transferrin, and glycolytic enzyme aldolase B. The AFP levels of Hep-Y1 and Hep-Y2 cells—detected using a commercial enzyme-linked immunosorbent assay—varied from days 1–3 dependent on growth conditions, with a peak level of 11.5 and 6.3 ng/mL, respectively. Western blot analysis of albumin, transferrin, and aldolase B were performed (Figure 3A). Albumin was strongly expressed in Hep-Y1, Hep-Y2, and HepG2 cells but not in 293-EBNA kidney cells. Transferrin, an iron-binding blood plasma glycoprotein that is mainly produced in the liver, was expressed by Hep-Y1, Hep-Y2, and HepG2 cells with increasing levels but not in 293-EBNA kidney cells. Aldolase B, a liver-type aldolase that played a key role in both glycolysis and gluconeogenesis, was strongly expressed in Hep-Y1 and HepG2 cells but weakly expressed in Hep-Y2 and 293-EBNA kidney cells.

**Figure 3:** Liver-specific protein expression in culture cells and HBV DNA detection in culture medium. (A) Expression of liver-specific proteins in Hep-Y1 and Hep-Y2 cells. Western blot analysis of albumin, transferrin, and aldolase B in Hep-Y1, Hep-Y2, HepG2, and 293-EBNA kidney cells. (B) PCR products in the medium of cultured Hep-Y1 cells and Hep-Y2 cells on a 2% agarose gel. M, molecular weight marker; P, PCR product from HBV DNA using the same PCR primers as positive control. Lanes 1 to 3, and lanes 4 to 6 were results of triplicate experiments.

### Detection of sustained HBV DNA in Hep-Y2 cells

The culture medium from both Hep-Y1 and Hep-Y2 cells were tested negative for HBsAg by either the enzyme immunoassay (Enzygnost HBsAg 5.0) or the radioimmunoassay (Ausria-II). To determine whether HBV replication was sustained in Hep-Y2 cells, a cell line derived from an occult HBV-infected patient, we assayed HBV DNA in the culture medium by PCR analysis. Figure 3B showed the presence of viral DNA in the medium of cultured Hep-Y2 cells. However, no viral DNA was detected in Hep-Y1 cells. HBsAg was negative in the culture medium of both cell lines. The intracellular HBV DNA level in Hep-Y1 cells was undetectable and in Hep-Y2 cells was 3.1719 × 10^6^ copies per 10^6^ cells, respectively.

### Permissiveness of HBV infection for Hep-Y1 and Hep-Y2 cells

Hep-Y1 and Hep-Y2 cells were found to share many morphological characteristics with normal human hepatocytes. Thus, we examined their susceptibility to HBV infection. To this end, we employed the same conditions that have previously been validated for in vitro infection of primary human hepatocytes [5]. Figure 4A showed the increasing levels of HBV DNA in culture medium from day 1 to 5 after HBV infection in Hep-Y1 cells by Southern blot analysis of the PCR amplicons. In contrast, HBV DNA was not detectable in normal serum (HBV-negative) infection.

**Figure 4:** HBV DNA replication in Hep-Y1 cells after HBV infection. (A) Southern blot kinetic analysis of PCR products after infection of Hep-Y1 cells with control normal HBV-negative serum and HBV-containing serum. P1 and P2, 1 pg and 50 pg of PCR products derived from HBV DNA were loaded. (B) Quantification of HBV DNA. The HBV-DNA levels in 10^6^ cells after HBV infection were measured by Cobas TaqMan HBV assay. D1-3, Day 1–3 after infection. 1 IU = 5.82 copies.

After HBV infection, the intracellular levels (cytoplasmic + extrachromosomal nuclear forms) of HBV DNA were also assessed by Cobas TaqMan HBV assays (Figure 4B). A progressively increasing HBV DNA level was observed in both Hep-Y1 and Y2 cells and the levels were higher when compared to those in HepG2 cells. Therefore, Hep-Y2 cells were also likely susceptible to HBV infection. To verify this point, we employed Southern blot analysis to compare the levels of HBV DNA produced in the cytosol after HBV infection. Cells were fractionated into cytoplasmic and nuclear fractions followed by Hirt's extraction. In Hep-Y1 cells, replicate intermediates of HBV DNA were detectable in the cytosol on day 5 after HBV infection by southern blot, confirming the permissiveness of HBV infection (Figure 5A).

**Figure 5:** Permissiveness of Hep-Y2 and Hep-Y1 cells for HBV infection. (A) Southern blot kinetic analysis of cytosolic and nuclear HBV DNA after infection of Hep-Y2 cells with control normal serum and HBV-containing serum. (B) Southern blot kinetic analysis of cytosolic and nuclear HBV DNA after infection of Hep-Y1 cells with control normal serum and HBV-containing serum. C, un-infected HepG2 cells as negative control. P, 20 pg of PCR product from HBV DNA as positive hybridization control.

In Hep-Y2 cells, southern blot analysis showed that extrachromosomal HBV DNA was detected in the nuclear but not cytoplasmic fractions even when control (HBV-negative) serum was used for infection (Figure 5B). This free form of HBV DNA was maintained in the nuclear fractions before and after day 9 of HBV infection, consistent with the status of occult HBV infection. Interestingly, replication intermediates of HBV DNA were detected in the cytosol on day 5 after HBV infection, which decreased gradually from day 5 to 9, suggesting permissiveness of HBV infection in Hep-Y2 cells (Figure 5B). Two species of HBV replication intermediates were discernable in Figure 5. The upper band corresponded to the relaxed circular form and the lower band corresponded to the double stranded linear form. The single stranded form and cccDNA were not seen in this study.

HBV DNA levels in the culture medium of infected Hep-Y2 cells were 26.4, 68.1, 388.2, and 32.8 ×10^4^ copies/mL at D3, D5, D7, and D9, respectively. HBV DNA level in the culture medium of infected Hep-Y1 cells was 280 copies/mL on D5 but was undetectable in D3, D7, and D9. HBeAg in the medium was negative in both cell lines after infection (D3 to 9). HBsAg in the medium was 1.46, 2.67, 3.24, and 2.89 IU/mL (D3, 5, 7, 9 after infection) in Hep-Y1 cells and 2.10, 3.54, 3.71 and 0.98 IU/mL (D3, 5, 7, 9 after infection) in Hep-Y2 cells using a quantification assay.

Immunofluorescence analysis was performed for Hep-Y1 and Y2 cells after HBV infection using a polyclonal anti-HBc (hepatitis B core) antibody (Figure 6) and anti-HBs antibody (Figure 7). Prominent cytoplasmic HBsAg and nuclear HBcAg expressions were detected in both Hep-Y1 and Y2 cells after infection. The infected cells ranged from 75 to 95% among independent experiments. These results indicated that Hep-Y1 and Y2 cells were efficiently infected by HBV.

**Figure 6:** Immunofluorescence analysis of core protein expression after HBV infection. (A) HBV-infected HepG2 and Hep-Y1 cells (left two panels) and HBV-negative serum inoculated Hep-Y1 and Hep-Y2 cells (right two panels, as negative controls) (B) HBV infected Hep-Y2 cells. Data of three independent experiments were shown (top to bottom). A polyclonal anti-HBc antibody was used to detect HBcAg. Nuclei were visualized by DAPI staining.

**Figure 7:** Immunofluorescence analysis of surface protein expression after HBV infection. (A) HBV-infected HepG2, Hep-Y1, and Hep-Y2 cells. (B) HBV-negative serum inoculated Hep-Y1 and Hep-Y2 cells. A polyclonal anti-HBs antibody was used to detect HBsAg. Nuclei were visualized by DAPI staining.

## Discussion

In this study, we established 2 HCC-derived cell lines, Hep-Y1 and Hep-Y2 cells. They maintained hepatocyte-like morphology as revealed by phase-contrast and transmission electron microscopy. Furthermore, optimal liver-specific functions such as the production of AFP, albumin, transferrin, and aldolase B were also observed. Similar to HepG2 cells, Hep-Y1 and Hep-Y2 cells were susceptible to HBV infection after treated with 2% DMSO. After infection with HBV-containing serum, HBcAg and HBsAg in Hep-Y1 and Hep-Y2 cells were detectable by immunofluorescence analysis. Compared with Hep-Y1 and Hep-Y2 cells, HepG2 cells infected with HBV produced much weaker immunofluorescence signals and lower HBV DNA levels. Hence, Hep-Y1 and Hep-Y2 cells seemed to be more susceptible to HBV infection than HepG2 cells. However, comparison between Hep-Y1, Hep-Y2, and another HBV-susceptible cell line—Hepa RG cells—has not been done in this study. Judging from the published data for Hepa RG cells, the HBV replication level in this cell line was even higher.

Occult HBV infection is defined as the persistence of viral genomes in the liver tissue—and, in some cases, also in the serum—of HBsAg-negative individuals [12]. The efficient eradication as well as monitoring of occult HBV infection is still a challenge in modern medicine. The Hep-Y2 cells, which were derived from an occult HBV infected patient, showed a phenotype consistent with occult HBV infection. To our knowledge, this is the first report of an occult hepatitis B-derived cell line carrying persistent extrachromosomal HBV DNA. In addition, this cell line is permissive for further exogenous HBV infection, a property never been observed before. Several issues could be explored by use of this cell line in the future. For example, how the nuclear HBV DNA in Hep-Y2 cells is maintained? Is there HBV DNA integration in the chromosome? Is there a complete HBV replication cycle in Hep-Y2 cells? Is there complete virion secretion? Is there S gene mutation? Several important experiments in the future are required to solve these puzzles. Previous reports have indicated that in growing cells, replication intermediates of HBV mostly located in the cytosol. However, in quiescent cells (G0/G1 phase), HBV DNA could accumulate in the nuclei [24], [25]. Presumably, this is caused by cell cycle regulation of nuclear transport for HBV core proteins [26]. In Hep-Y2 cells, however, a nuclear form of HBV DNA was maintained in growing cells. Conceivably, some unknown host and viral factors are involved.

The serum sample from the occult HBV infected patient (from whom Hep-Y2 cells were derived) was negative for HBV DNA, whereas the aspirated liver cells were positive for HBV DNA. As such, we were unable to obtain the “initial” strain of HBV for comparison because of insufficient amount of tissue sample. In Hep-Y2 cells, partial HBV genome derived from the extrachromosomal nuclear form was cloned and sequenced. However, there remained a gap of around 1000 bp between the core and pre-S coding regions (data not shown). Presumably, this is caused by either deletion or recombination. Another important question to be asked was whether an integrated form of HBV genome existed in Hep-Y2 cells. These tissues should be clarified in future studies.

Occult HBV may have an important impact in several different clinical contexts, including the transmission of occult HBV infection by blood transfusion or organ transplantation and acute reactivation under immunosuppressive status. Moreover, evidence has suggested that it can enhance the progression of liver fibrosis and, above all, the development of HCC [12]. Accordingly, how to adequately detect and treat occult HBV infection is an important issue, which is still unclear at this time. By use of Hep-Y2 cells, we may be able to identify more effective and accurate therapeutic strategies with the presently available antiviral agents, which include nucleot(s)ide analogs and interferon.

In summary, we established Hep-Y1 and Hep-Y2 hepatoma cell lines which were permissive for HBV infection after DMSO treatment. Furthermore, Hep-Y2 cells retained the phenotype of occult HBV infection and maintained an extrachromosomal form of persistent HBV DNA in the nuclei. Therefore, these cell lines serve as important tools for further studies on HBV host–pathogen interaction. Additionally, Hep-Y2 cells provide a powerful tool for investigating the molecular virology of occult HBV infection.
